The article "Exosomal miR-128-3p Promotes Epithelial-to-Mesenchymal Transition in Colorectal Cancer Cells by Targeting FOXO4 via TGF-β/SMAD and JAK/STAT3 Signaling" was retracted in 2024. Reasons: unreliable data; unreliable results or conclusions; concerns about the images.

# Exosomal miR-128-3p Promotes Epithelial-to-Mesenchymal Transition in Colorectal Cancer Cells by Targeting FOXO4 via TGF-β/SMAD and JAK/STAT3 Signaling

**DOI:** 10.3389/fcell.2021.568738

**Published:** 2021-02-09

**Authors:** Jian Bai, Xue Zhang, Dongdong Shi, Zhenxian Xiang, Shuyi Wang, Chaogang Yang, Qing Liu, Sihao Huang, Yan Fang, Weisong Zhang, Jialin Song, Bin Xiong

**Affiliations:** ^1^Department of Gastrointestinal Surgery & Department of Gastric and Colorectal Surgical Oncology, Zhongnan Hospital of Wuhan University, Wuhan, China; ^2^Department of Anesthesiology, Peking University Third Hospital, Beijing, China; ^3^Hubei Key Laboratory of Tumor Biological Behaviors, Wuhan, China; ^4^Hubei Cancer Clinical Study Center, Wuhan, China; ^5^Department of General Practice, Beijing Friendship Hospital, Capital Medical University, Beijing, China; ^6^Department of Radiation Oncology and Medical Oncology, Zhongnan Hospital of Wuhan University, Wuhan, China

**Keywords:** microRNA, EMT, extracellular vesicle, molecular signaling, gastrointestinal

## Abstract

Epithelial-to-mesenchymal transition (EMT) is a key process that occurs during tumor metastasis, affecting a variety of malignancies including colorectal cancer (CRC). Exosomes mediate cell-cell communication by transporting cell-derived proteins and nucleic acids, including microRNAs (miRNAs). Exosomal delivery of miRNAs plays an important role in tumor initiation, development, and progression. In this study, we investigated the effect of exosomal transfer between CRC cells and aimed to identify specific miRNAs and downstream targets involved in EMT and metastasis in CRC cells. High expression of miR-128-3p was identified in exosomes derived from EMT-induced HCT-116 cells. Altered miR-128-3p expression in CRC cells led to distinct changes in proliferation, migration, invasion, and EMT. Mechanistically, miR-128-3p overexpression downregulated the expression of FOXO4 and induced the activation of TGF-β/SMAD and JAK/STAT3 signaling in CRC cells and xenografted tumors, which led to EMT. Clinically, high expression of miR-128-3p was significantly associated with perineural invasion, lymphovascular invasion, tumor stage, and CA 19-9 content in CRC patients. We revealed that exosomal miR-128-3p regulates EMT by directly suppressing its downstream target gene FOXO4 to activate TGF-β/SMAD and JAK/STAT3 signaling, and the properties of the miR-128-3p/FOXO4 axis were horizontally transferred via exosomal delivery. In turn, exosomal miR-128-3p could be considered as a new therapeutic vehicle for CRC.

## Introduction

Colorectal cancer (CRC) is the third most common cancer worldwide, and metastasis and invasion are the leading causes of mortality in CRC patients (Smith et al., 2015). Intrinsic mechanisms and extrinsic factors influence tumor development and aggressiveness. A growing body of evidence has reported the critical role of epithelial-to-mesenchymal transition (EMT) in cancer metastasis and invasion by endowing tumor cells with a motile and invasive phenotype (Ma et al., 2017; Zhao et al., 2017). EMT induces the transformation of epithelial cells into mesenchymal cells, promoting cell movement, metastasis, and cancer progression (Pradella et al., 2017; Suarez-Carmona et al., 2017). However, the underlying molecular mechanisms that regulate metastasis and invasion are not well-studied. Further understanding of the metastatic mechanisms of CRC may greatly improve the poor survival of CRC patients.

Multiple factors are involved in the initiation and progression of EMT, such as abnormal cytokine pathways, tumor-stromal cell interaction, and hypoxia (Shi et al., 2014). Signaling pathways such as transforming growth factor-beta/small mothers against decapentaplegic (TGF-β/SMAD), Notch/nuclear factor-κB, and Wnt/glycogen synthase kinase 3β are involved in tumor EMT (Zhou and Hung, 2005; Fender et al., 2015; Ouanouki et al., 2017). In addition, inflammatory factors can promote tumor growth and induce EMT in a variety of malignancies, including breast, liver, head and neck, and colorectal tumors via the regulation of Janus kinase/signal transducer and activator of transcription 3 (JAK/STAT3) and TGF-β signaling (Sehgal, 2010; Crusz and Balkwill, 2015). Inflammatory mediators in the tumor microenvironment coordinate a series of inflammatory responses that act on both malignant and non-malignant cells in the form of autocrine or paracrine signaling (Sehgal, 2010). For example, interleukin (IL)-6, an inflammatory cytokine, is a potent inducer of EMT in a variety of cancers including breast cancer (Gyamfi et al., 2018), cervical carcinoma (Miao et al., 2014), and colon cancer (Kang et al., 2018).

Cellular crosstalk occurring during physiological processes such as tumorigenesis and EMT take place via intercellular messenger particles, of which exosomes have recently gained wide attention. Exosomes are extracellular vesicles with diameters ranging from 30 to 100 nm that are released from normal and tumor cells and represent an intercellular communication route (Simons and Raposo, 2009). Exosomal secretion is reportedly increased in tumor cells and has immunosuppressive effects, which maintain tumor survival and development by inducing tumor growth, invasion, angiogenesis, and metastasis (Riches et al., 2014). Effectors delivered by exosomes, including transcription factors, non-coding regulatory RNAs, oncogenes, and mRNAs, are transferred into recipient cells by endocytosis (Barile and Vassalli, 2017). Among the contents of exosomes, microRNAs (miRNAs) have been shown to govern important processes that contribute to the pathophysiological consequences of CRC (Li et al., 2017). miRNAs control gene expression and signal activation involved in various physiological and pathological processes (Elsharawy et al., 2016; Fang et al., 2017; Yang et al., 2017). Recent studies have shown that miRNAs play a critical role in tumor invasion and metastasis by regulating EMT (Beermann et al., 2016; Zhang et al., 2016). Li et al. reported that the long non-coding RNA XIST promoted TGF-β-induced EMT, cell invasion, and metastasis by regulating miR-367/miR-141 in non-small-cell lung cancer (Li et al., 2018). The number of verified miRNAs is constantly growing, and recent research has focused on the value of miRNAs especially in metastatic CRC. Gaedcke et al. identified at least 49 distinct miRNAs that are significantly expressed in rectal cancer, out of which 28 were already described for CRC (Gaedcke et al., 2012). These regulatory miRNAs provide new targets and directions for the clinical treatment of tumors and prognosis improvement. In terms of CRC, the effect of exosomes in regulating the progression and growth of colorectal tumors remains unclear.

In this study, we explored and verified the mechanism of CRC-derived exosomal miRNAs in the process of EMT. We first induced EMT in HCT-116 cells using IL-6 and identified differentially expressed miRNAs in exosomes derived from IL-6-induced and non-induced cells. The effect of differentially expressed miRNAs on EMT in HCT-116 cells and colorectal tumor progression was investigated *in vitro* and *in vivo*, respectively.

## Materials and Methods

### Cell Culture and Exosome Isolation

The human CRC cell lines HCT-116 and SW480 were purchased from the Cell Bank of the Chinese Academy of Sciences (Shanghai, China). HCT-116 cells were cultured in RPMI 1640 medium (Gibco, USA) and SW480 cells were cultured in L15 medium (LA9510, Solarbio, Beijing, China), both supplemented with 10% (v/v) fetal bovine serum (FBS), 10 U/mL penicillin, and 100 mg/mL streptomycin (Gibco, Carlsbad, CA) at 37°C with 5% CO_2_. For IL-6 induction, the cells were treated with 100 ng/mL IL-6 for 48 h. Exosomes were isolated from HCT-116 cells as previously described (Thery et al., 2006). The cell culture medium (50 mL) was harvested after 3 days and centrifuged at 300 × g for 10 min, 2,000 × g for 10 min, and 10,000 × g for 30 min to remove residual cells and debris. After ultracentrifugation twice at 100,000 × g for 70 min (Ultracentrifuge, Optima L-100 XP, Beckman Coulter), the cell pellet was collected and resuspended in 50–100 mL of phosphate-buffered saline (PBS). The isolation of serum exosomes was performed using the Exosome Isolation kit (SBI).

### PKH67 Staining for Exosome Uptake Evaluation

Exosomes were fluorescently labeled using the PKH67 Green Fluorescent Cell Linker Midi Kit (MIDI67-1KT, Sigma-Aldrich, St. Louis, MO). After ultracentrifugation, 10 μg of exosomes were mixed with 1 mL of diluent with 4 μL of PKH67 reagent included in the kit. The exosomes were incubated for 4 min and excess dye was removed with 2 mL of 0.5% bovine serum albumin in PBS. The labeled exosomes were ultracentrifuged at 100,000 × g and washed twice to remove the remaining dye. HCT-116 cells were seeded in a 24-well plate at 1 × 10^4^ cells/well at 37°C in 5% CO_2_. After 12 h of culture, 10 μg of fluorescently labeled exosomes diluted in 100 μL of PBS were added to each well, and photos were taken under a fluorescence microscope after 2 and 24 h.

### miRNA Array and Bioinformatic Analysis

RNA was extracted from exosomes derived from non-induced and IL-6-induced HCT-116 cells for microarray analysis. The microarray experiments were carried out commercially by Allwegene Technologies (Beijing, China) following standard Agilent protocols. Differentially expressed miRNAs were screened from exosome libraries. Based on miRNA analysis and previous literature, miR-128-3p was selected for the subsequent studies. According to the miRDB web site (http://www.mirdb.org/cgi-bin/search.cgi), miRNA target genes were screened.

### Transmission Electron Microscopy (TEM)

For morphological investigation using TEM, 3 μL of exosome pellet was placed on formvar carbon-coated 200-mesh copper electron microscopy grids. The specimen was incubated for 5 min at room temperature and subjected to standard uranyl acetate staining. The grid was washed three times with PBS and allowed to semi-dry at room temperature before TEM observation (Hitachi H7500 TEM, Tokyo, Japan).

### Plasmid Construction and Transfection

Overexpression vectors and interference vectors (siRNA) for forkhead box protein O4 (FOXO4) were chemically synthesized, constructed, sequenced, and identified by Wuhan Myhalic Biotechnological Co., Ltd. (Wuhan, China) with the following sequences: FOXO4 overexpression forward, 5′-TTGCGGCCGCATGGATCCGGGGAATGAGAAT-3′, reverse 5′-GCTCTAGATCAGGGATCTGGCTCAAAGTT-3′; FOXO4 interference, 5′-GCGGAGGAAATACCAGCTTCA-3′. HCT-116 cells were transfected with overexpression or interference vectors using Lipofectamine 2000 following the manufacturer's instructions. miR-128-3p mimics and inhibitors (and corresponding negative controls, NC) were obtained from Wuhan Myhalic Biotechnological Co., Ltd. After 48 h of transfection, the cells were harvested for further assay or exosome isolation as described in the Cell Culture and Exosome Isolation section.

### Quantitative Reverse Transcription Polymerase Chain Reaction (qRT-PCR)

Total RNA was extracted from exosomes by SeraMir (System Biosciences) following the manufacturer's instructions and cellular RNA was extracted using the RNAprep pure cell/bacteria kit (TIANGEN, Beijing, China). The purity of the isolated RNA was determined at OD260/280 using a Nanodrop ND-1000 (Thermo Scientific), and integrity was assessed by 1% agarose gel electrophoresis. RNAs were reverse-transcribed to first-strand cDNA using the PrimeScipt RT Reagent Kit (TaKaRa, Dalian, China). The cDNA was subjected to qRT-PCR using the SYBR kit (TaKaRa, Dalian, China). miR-128-3p expression was quantified with a stem-loop real-time PCR miRNA kit (Ribobio, Guangzhou, China). The threshold cycle (Ct) was determined for each reaction using the 2^−ΔΔCt^ method, and the expression of each gene of interest was normalized to that of the endogenous control gene (U6 for miRNAs or GAPDH for mRNAs). The primer sequences in the study are shown in Supplementary Table 1.

### Luciferase Reporter Assay

HCT-116 cells were co-transfected with 500 ng of wild-type (WT) or mutant (MUT) 3′-untranslated region (UTR) of FOXO4 and 50 nM miR-128-3p mimics or 100 nM miR-128-3p inhibitors using Lipofectamine 2000 (Invitrogen, USA) following the manufacturer's instructions. After 48 h, the cells were lysed using the Dual-Luciferase Reporter Assay System (Promega, Madison, WI, USA), and luciferase activity was measured using a GloMax20/20 Luminometer (Promega). Luciferase activity was normalized by renilla/firefly luciferase signal in HCT-116 cells. WT and MUT 3′-UTR segments were prepared as follows: FOXO4 222–228 WT, 5′-CTAGCGATGGGAGGGGAAAGGGGAGAGGGTTTTTCTCACTGTGCCAATTAGGGGGTAAGGCCCCCTCTCA-3′; MUT, 5′-CTAGCGATGGGAGGGGAAAGGGGAGAGGGTTTTTCTCTTGCAGCCAATTAGGGGGTAAGGCCCCCTCTCA-3′.

### RNA Stability Assessment

To evaluate the effect of miR-128-3p on the stability of FOXO4 RNA, HCT-116 cells were transfected for 48 h with mimics of miR-128-3p or their negative control (NC) in 6-well plates as described in the Plasmid Construction and Trasfection section. Thereafter, actinomycin D (abs810015, absin, Shanghai, China) was added to each well at 5 μg/mL and the plate was incubated for 0, 2, 4, 8, and 16 h. At the end of the incubation period, RNA was extracted from the cells and the mRNA expression of FOXO4 was evaluated by PCR as described in the Quantitative Reverse Transcription Polymerase Chain Reaction (qRT-PCR) section.

### Cell Counting Kit (CCK)-8 Assay

Cells were seeded into a 96-well plate at 5 × 10^3^ cells per well and 10 μL of CCK-8 reagent (Bio-swamp, Wuhan, China, PAB180031) was added to each well. After 4 h of incubation at 37°C, the absorbance of the wells was measured using a microplate reader (Sunrise Microplate Reader, TECAN, Switzerland) at 450 nm.

### Western Blot

A total of 30 μg of protein was resuspended in sodium dodecyl sulfate (SDS) sample buffer and boiled for 5 min. Equal amounts of protein were separated by 10% SDS-polyacrylamide gel electrophoresis (Sigma-Aldrich), followed by electrotransfer to polyvinylidene difluoride membranes (Sigma-Aldrich). The membranes were incubated with blocking buffer (Sigma-Aldrich) for 1 h at room temperature and with primary antibodies against CD63 (1:1,000, ab134045, abcam), CD81 (1:1,000, ab109201, abcam), TSG101 (1:1,000, ab125011, abcam), FOXO4 (1:1,000, ab63254, abcam), suppressor of cytokine signaling 5 (SOCS5, 1:2,000, PAB35610, Bio-swamp, Wuhan, China), APC membrane recruitment protein 2 (AMER2, 1:1,000, PA5-71433, Thermo), hypermethylated in cancer 1 (HIC1, 1:2,000, PAB36143, Bio-swamp), SMAD-specific E3 ubiquitin protein ligase 2 (SMURF2, 1:1,000, ab94483, abcam), TGF-β (1:2,000, PAB33215, Bio-swamp), SMAD2 (1:2,000, PAB30712, Bio-swamp), SMAD3 (1:2,000, PAB30705, Bio-swamp), p-JAK2 (1:2,000, PAB43391-P, Bio-swamp), JAK2 (1:2,000, PAB30711, Bio-swamp), p-JAK-3 (1:2,000, PAB43511-P, Bio-swamp), JAK-3 (1:2,000, PAB30209, Bio-swamp), p-STAT3 (1:2,000, PAB36336-P, Bio-swamp), STAT3 (1:500, PAB30641, Bio-swamp), E-cadherin (1:1,000, PAB30714, Bio-swamp), ZO-1 (1:1,000, PAB43761, Bio-swamp), vimentin (1:1,000, PAB30692, Bio-swamp), N-cadherin (1:1,000, PAB33543, Bio-swamp), and GAPDH (1:2,000, PAB36264, Bio-swamp) at 4°C overnight. Then, the membranes were washed with Tris-buffered saline and incubated in goat anti-rabbit IgG antibody (1:20,000, PAB160011, Bio-swamp) for 2 h at room temperature. Immunoreactivity was visualized by colorimetric reaction using an enhanced chemiluminescence substrate buffer (Millipore, MA, USA). Membranes were scanned with Gel Doz EZ imager (Bio-rad, CA, USA).

### Wound Healing Assay

The cells were cultured in 6-well plates overnight. The cell monolayers were wounded by scratching with a plastic 10-μL micropipette tip and washed twice with PBS. Fresh FBS-free growth medium was added to the plates. Images of the scratched gap were photographed using a microscope at 0 and 48 h. Gap width was measured using ImageJ.

### Transwell Assay

Medium containing 10% FBS was added to the lower Transwell chambers and the upper chambers were covered with a mixture of RPMI-1640 and Matrigel (BD Biosciences, San Jose, CA). Cells were transfected as described above for 48 h and seeded in the upper chamber of Transwell plates (Corning, NY, USA) with FBS-free medium. Cells remaining on the top of the chambers were removed with cotton swabs, while those that went through the membrane were stained with 0.5% crystal violet (Sigma-Aldrich), observed, and counted under a microscope.

### Xenograft Assays

All animal experiments were performed in accordance with the “Guidelines for Animal Care and Use of the Model Animal Research Institute at Wuhan Myhalic Biotechnology Co., Ltd.” and were approved by the Institutional Review Board (approval number HLK-20181031-02). Thirty BALB/c nude mice (female, 4–6 weeks of age, weighing 16–20 g) were purchased from Beijing Vital River Laboratory Animal Technology Co., Ltd. (Beijing, China). Each mouse was subcutaneously injected with 5 × 10^6^ HCT-116 cells on the right flank region. After 3 days, the transplanted mice were randomly divided into six groups (*n* = 5 per group). Mice in the model group (Mod) were injected with 50 μL of PBS. For exosome treatment, exosomes (from non-transfected HCT-116 cells or those transfected with miR-128-3p overexpression vectors, miR-128-3p interference vectors, or the corresponding negative controls) were directly injected into the mice at 10 μg exosomes/50 μL of PBS. Tumor dimensions were measured at the indicated time points. After 21 days, tumor volume was calculated and the tumors were collected for further experiments.

### Patients and Serum Samples

Serum samples were acquired from 66 patients diagnosed with primary CRC at Zhongnan Hospital of Wuhan University (Wuhan, China). All samples were collected with informed consent, and all related procedures were performed with the approval of the internal review and ethics boards of Zhongnan Hospital of Wuhan University. The enrolled patients were categorized into two groups based on the median score of exosomal miR-128-3p expression (identified as a differentially expressed miRNA by bioinformatic analysis): high expression: > median score; low expression: ≤ median score.

### Statistics Analysis

All statistical analyses were performed with SPSS statistical software (version 22.0, IBM SPSS, USA). Chi-square test and logistic regression analysis were applied to analyze the relationship between exosomal miR-128-3p expression and clinicopathological status. One-way analysis of variance was performed in experiments for cell cultures and xenograft assays. The results were expressed as the mean ± standard deviation from at least three independent experiments and P < 0.05 was considered statistically significant.

## Results

### IL-6 Induced EMT in HCT-116 Cells

IL-6, a well-known pro-inflammatory cytokine, is known to induce EMT in a variety of tumors including esophageal adenocarcinoma (Ebbing et al., 2019) and biliary tract cancer (Yamada et al., 2013). This results in the development of chemoresistance and metastasis, among other tumorigenic traits. To induce EMT in HCT-116 cells, we treated the cells with IL-6 at 100 ng/mL for 0, 48, or 72 h. We assessed the cell viability, invasion, and migration and the expression of the epithelial marker E-cadherin and mesenchymal markers ZO-1, vimentin, and N-cadherin. The results demonstrated that IL-6 significantly increased the viability and promoted the invasion and migration of HCT-116 cells (Figures 1A–C). Compared with the control group (absence of IL-6), E-cadherin expression was suppressed by IL-6, whereas ZO-1, vimentin, and N-cadherin were significantly upregulated in HCT-116 cells (Figure 1D). These results indicated that in response to IL-6 exposure, EMT took place in HCT-116 cells. In addition, IL-6 induced the activation of TGF-β/SMAD and JAK/STAT3 signaling via the upregulation of TGF-β, SMAD2, SMAD3, p-JAK, and p-STAT3 (Figures 1E,F).

**Figure 1:** IL-6 induced EMT in HCT-116 cells via TGF-β/SMAD and JAK/STAT3 signaling. **(A)** Cell viability was detected by CCK-8 assay. **(B)** Transwell invasion assay of HCT-116 cells. Total number of cells was counted manually in five fields, scale bar = 100 μm. **(C)** Wound healing assay and quantification of scratch gap width at 0 and 48 h, scale bar = 200 μm. **(D)** Western blot and quantification of the expression of EMT markers E-cadherin, ZO-1, vimentin, and N-cadherin in HCT-116 cells. Protein expression was normalized to that of GAPDH. **(E)** Western blot and quantification of the expression of TGF-β, SMAD2, and SMAD3 in HCT-116 cells. Protein expression was normalized to that of GAPDH. **(F)** Western blot and quantification of p-JAK2, JAK2, p-STAT3, and STAT3 in HCT-116 cells. Phosphorylated protein expression was normalized to that of total proteins. Data are shown as the mean ± SD (*n* = 3); *P < 0.05.

### IL-6 Induced EMT Is Correlated With Exosomal miR-128-3p via FOXO4 Targeting

The morphology and phenotype of vesicles isolated from normal and IL-6-induced HCT-116 cells were identified based on the characteristics of exosomes. Morphological observation by TEM (Figure 2A) revealed that the isolated vesicles possessed a double-layer membrane structure with diameters of approximately 40–100 nm. Exosomal markers CD63, CD81, and TSG101 were detected in the vesicles, whereas only minimal expression was detected in the cell lysate (Figure 2B). Collectively, these observations confirmed that the vesicles isolated in our experiments were exosomes.

**Figure 2:** Characterization of exosomes derived from CRC cells. **(A)** TEM images showing small vesicles of ~40–100 nm in diameter, scale bar = 100 nm. **(B)** Western blot characterization of exosomal markers CD63, CD81, and TSG101 in isolated exosomes and cell lysates after extraction. **(C)** Heat map showing the changes in miRNA expression in exosomes isolated from non-induced (Con) and IL-6-induced HCT-116 cells. **(D)** qRT-PCR of exosomal miRNA expression in non-induced (Con) and IL-6-induced HCT-116 cells. **(E)** qRT-PCR and **(F)** western blot of the expression of miR-128-3p target genes FOXO4, SOCS5, AMER2, HIC1, and SMURF2 in non-induced (Con) and IL-6-induced HCT-116 cells. Protein expression was normalized to that of GAPDH. **(G)** Relative luciferase activity of reporter plasmids carrying WT or MUT FOXO4 3′-UTR in HCT-116 cells co-transfected with miR-128-3p mimics or its negative control (miR-NC). **(H)** Decay curve representative of FOXO4 mRNA degradation in HCT-116 cells carrying miR-128-3p mimics or mimic-NC. Data are shown as the mean ± SD (*n* = 3); *P < 0.05.

High-throughput sequencing was performed to analyze the differentially expressed miRNAs in exosomes from normal and IL-6-induced HCT-116 cells (Figures 2C,D). Among the identified miRNAs, 13 were upregulated and three were downregulated in IL-6-induced HCT-116 cells compared to those in normal HCT-116 cells (Supplementary Table 2). Based on miRNA analysis and previous literature, miR-128-3p was selected for the subsequent studies. According to the miRDB web site, five genes (FOXO4, SOCS5, AMER2, HIC1, and SMURF2) were identified as targets of miR-128-3p. The mRNA and protein expression of these targets were detected in normal and IL-6-induced HCT-116 cells (Figures 2E,F), revealing that FOXO4, SOCS5, AMER2, HIC1, and SMURF2 were downregulated by IL-6 at both the gene and protein level. Based on previous reports on the role of FOXO4 as a tumor suppressor gene by inhibiting tumor proliferation and metastasis (Su et al., 2014), FOXO4 was selected as the target gene for miR-128-3p in this study.

To confirm the direct regulation of FOXO4 expression by miR-128-3p, the dual-luciferase reporter assay was carried out. WT luciferase reporter vectors carrying the FOXO4 3′-UTR sequence or MUT reporter vectors carrying point mutations of the putative miR-128-3p binding sites were co-transfected with miR-128-3p mimics or negative controls (miR-NC), separately. The results indicated that miR-128-3p inhibited luciferase activity in WT FOXO4 3′-UTR-transfected HCT-116 cells, whereas it did not influence luciferase activity in cells carrying mutant FOXO4 3′-UTR (Figure 2G), suggesting that miR-128-3p binds directly to the 3′-UTR of FOXO4. We further analyzed the stability of FOXO4 mRNA by transfecting HCT-116 cells with miR-128-3p mimics or miR-NC and detecting the mRNA expression of FOXO4 at designated time points (Figure 2H). With time, the degree of FOXO4 mRNA degradation in the presence of miR-128-3p mimics was significantly greater than that induced by miR-NC, suggesting that the mechanism through which miR-128-3p regulates FOXO4 is the direct targeting of mRNA stability.

### miR-128-3p Induced EMT and Promoted CRC Cell Migration and Invasion via FOXO4 Silencing

To clarify the role of miR-128-3p and FOXO4 in EMT, HCT-116 cells were transfected with overexpression or interference vectors for miR-128-3p or FOXO4, with corresponding negative controls (NC). The expression of miR-128-3p and FOXO4 mRNA was detected by qRT-PCR (Figures 3A–C), confirming successful transfection. Note in particular that miR-128-3p overexpression significantly downregulated the mRNA expression of FOXO4 in HCT-116 cells (Figure 3B). miR-128-3p overexpression and FOXO4 interference significantly increased cell viability (Figures 3D,E), migration (Figures 3F,G), and invasion (Figures 3H,I). Furthermore, miR-128-3p overexpression and FOXO4 interference promoted EMT by downregulating E-cadherin and upregulating ZO-1, vimentin, and N-cadherin (Figure 4A), while the TGF-β/SMAD and JAK/STAT3 signaling pathways were activated via the upregulation of TGF-β, SMAD2, SMAD3, p-JAK2/3, and p-STAT3 in HCT-116 cells (Figures 4B,C). Conversely, CRC cell viability, migration, invasion, EMT, and TGF-β/SMAD and JAK/STAT3 activation were inhibited by miR-128-3p interference and FOXO4 overexpression. Taken together, these results demonstrated the effect of miR-128-3p in promoting CRC progressing via its suppression of FOXO4.

**Figure 3:** Upregulation of miR-128-3p and downregulation of FOXO4 induced EMT in CRC cells. qRT-PCR of **(A)** miR-128-3p and **(B)** FOXO4 mRNA expression in HCT-116 cells transfected with miR-128-3p overexpression or interference vectors (or corresponding NC). **(C)** qRT-PCR of FOXO4 mRNA expression in HCT-116 cells transfected with FOXO4 overexpression or interference vectors (or corresponding NC). CCK-8 detection of the viability of HCT-116 cells after transfection with overexpression or interference vectors (or corresponding NC) of **(D)** miR-128-3p and **(E)** FOXO4. Wound healing assay (scale bar = 200 μm) after HCT-116 cells were transfected with overexpression or interference vectors (or corresponding NC) of **(F)** miR-128-3p and **(G)** FOXO4. Transwell invasion assay (scale bar = 100 μm) after HCT-116 cells were transfected with overexpression or interference vectors (or corresponding NC) of **(H)** miR-128-3p and **(I)** FOXO4. Data are shown as the mean ± SD (*n* = 3); *P < 0.05.

**Figure 4:** miR-128-3p overexpression and FOXO4 interference regulated the expression of EMT markers and TGF-β/SMAD and JAK/STAT3 signaling. HCT-116 cells were transfected with overexpression or interference vectors (or corresponding NC) of miR-128-3p or FOXO4. **(A)** Western blot and quantification of EMT markers E-cadherin, ZO-1, vimentin, and N-cadherin in HCT-116 cells. Protein expression was normalized to that of GAPDH. **(B)** Western blot and quantification of TGF-β, SMAD2, and SMAD3 in HCT-116 cells. Protein expression was normalized to that of GAPDH. **(C)** Western blot and quantification of p-JAK2, JAK2, p-JAK3, JAK3, p-STAT3, and STAT3 in HCT-116 cells. Phosphorylated protein expression was normalized to that of total proteins. Data are shown as the mean ± SD (*n* = 3); *P < 0.05.

To further confirm the role of FOXO4, rescue assays were performed by co-transfecting CRC cells with miR-128-3p and FOXO4 interference or overexpression vectors. The expression of miR-128-3p and the mRNA and protein expression of FOXO4 in HCT-116 cells were detected by qRT-PCR and western blot, respectively (Figures 5A–C). In terms of cell behavior and EMT properties, CRC cell migration was significantly enhanced by miR-128-3p overexpression (Figure 5D), whereas EMT was promoted as demonstrated by the downregulation of E-cadherin and upregulation of ZO-1, vimentin, and N-cadherin (Figure 5E). However, FOXO4 overexpression reversed the enhancement in migration and EMT caused by miR-128-3p in CRC cells, suggesting that the effect of miR-128-3p was dependent on its regulation of FOXO4.

**Figure 5:** FOXO4 inhibited miR-128-3p-induced EMT in CRC cells. HCT-116 cells were transfected with overexpression or interference vectors of miR-128-3p and/or FOXO4. qRT-PCR of **(A)** miR-128-3p expression and **(B)** FOXO4 mRNA expression in HCT-116 cells. **(C)** Western blot and quantification of FOXO4 protein expression in HCT-116 cells. Protein expression was normalized to that of GAPDH. **(D)** Western blot and quantification of EMT markers E-cadherin, ZO-1, vimentin, and N-cadherin in HCT-116 cells. Protein expression was normalized to that of GAPDH. **(E)** Wound healing assay, scale bar = 200 μm. Data are shown as the mean ± SD (*n* = 3); *P < 0.05.

### Exosomal miR-128-3p Induced EMT in HCT-116 Cells

To examine whether the effect of miR-128-3p is transferrable between cells via exosomes, we co-cultured HCT-116 cells with exosomes isolated from normal HCT-116 cells (Control-Exo) or from HCT-116 cells subjected to miR-128-3p overexpression (miR-128-3p-Exo) or interference (si-miR-Exo), with corresponding negative controls (miR-128-3p-NC-Exo and si-miR-NC-Exo, respectively). Prior to co-culture, the relative expression of miR-128-3p was detected in the isolated exosomes (Figure 6A). Exosome uptake by HCT-116 cells was confirmed by PKH67 staining at 2 and 24 h of co-culture (Figure 6B), and the evident increase in green fluorescence is indicative of gradual exosome endocytosis over time (only the results for Control-Exo are shown). The expression of miR-128-3p (Figure 6C) and FOXO4 mRNA (Figure 6D) in exosome-treated HCT-116 cells were detected, confirming that the effect of transfection was horizontally transferred by exosomes. In addition, exosomes isolated from miR-128-3p-overexpressing HCT-116 cells significantly enhanced cell viability (Figure 6E), migration (Figure 6F), and invasion (Figure 6G), while downregulating E-cadherin, upregulating ZO-1, vimentin, and N-cadherin (Figure 7A), and activating TGF-β/SMAD (Figure 7B) and JAK/STAT3 (Figure 7C) signaling. The abovementioned experiments evaluating miR-128-3p and FOXO4 mRNA expression, cell viability, migration, and invasion were performed in another CRC cell line (SW480) in parallel. Notably, the behavior of SW480 cells co-cultured with HCT-116-derived exosomes was similar to that of HCT-116 cells (Supplementary Figure 1), suggesting that the effect of miR-128-3p is transferrable to different CRC cell types via exosomal delivery.

**Figure 6:** Co-culture of HCT-116 cells with exosomes isolated from HCT-116 cells. HCT-116 cells were co-cultured with exosomes that were isolated from HCT-116 cells transfected with overexpression or interference vectors (or corresponding NC) of miR-128-3p. **(A)** qRT-PCR of relative expression of miR-128-3p in exosomes isolated from HCT-116 cells. **(B)** Indication of exosome uptake after 2 and 24 h in HCT-116 cells by fluorescence staining of PKH67. Green fluorescence represents PKH-labeled exosomes and blue fluorescence represent the cell nuclei. Scale bar = 50 μm. qRT-PCR of **(C)** miR-128-3p and **(D)** FOXO4 mRNA expression in HCT-116 cells co-cultured with exosomes. **(E)** Viability of HCT-116 cells was detected by CCK-8 assay after co-culture with exosomes. **(F)** Wound healing assay, scale bar = 200 μm. **(G)** Transwell invasion assay, scale bar = 100 μm. Data are shown as the mean ± SD (*n* = 3); *P < 0.05.

**Figure 7:** Exosomes isolated from miR-128-3p-overexpressing HCT-116 cells induced EMT in HCT-116 cells. HCT-116 cells were cultured with exosomes that were isolated from HCT-116 cells transfected with overexpression or interference vectors (or corresponding NC) of miR-128-3p. **(A)** Western blot and quantification of EMT markers E-cadherin, ZO-1, vimentin, and N-cadherin in HCT-116 cells. Protein expression was normalized to that of GAPDH. **(B)** Western blot and quantification of TGF-β, SMAD2, and SMAD3 in HCT-116 cells. Protein expression was normalized to that of GAPDH. **(C)** Western blot and quantification of p-JAK2, JAK2, p-JAK3, JAK3, p-STAT3, and STAT3 in HCT-116 cells. Phosphorylated protein expression was normalized to that of total proteins. Data are shown as the mean ± SD (*n* = 3); *P < 0.05.

### Exosomal miR-128-3p Induced Tumor Growth in Nude Mice

Nude mice xenografted with tumors induced by subcutaneous injection of HCT-116 cells were treated with tail vein injection of exosomes, and tumor growth was evaluated. Tumor growth was inhibited by exosomes isolated from si-miR-128-3p-transfected HCT-116 cells but promoted by those isolated from miR-128-3p-overexpressing cells (Figures 8A,B). Compared to xenografted animals treated with PBS (Mod), miR-128-3p-Exo significantly increased the expression of miR-128-3p (Figure 8C) and decreased that of FOXO4 mRNA (Figure 8D) in tumor tissues. In addition, the expression of E-cadherin was inhibited while that of ZO-1, vimentin, and N-cadherin was induced by miR-128-3p-overexpressing exosomes in tumor tissues (Figure 8E). Concurrently, miR-128-3p-overexpressing exosomes induced the activation of TGF-β/SMAD (Figure 8F) and JAK/STAT3 (Figure 8G) in tumor tissues, but exosomes isolated from miR-128-3p-silenced HCT-116 cells (si-miR-128-3p-Exo) inhibited tumor growth, likely by enhancing the expression FOXO4.

**Figure 8:** Exosomes isolated from miR-128-3p-overexpressing HCT-116 cells induced tumor growth in nude mice. **(A)** Tumors isolated at the end of experimental period. **(B)** Tumor growth curve showing tumor volume over time. qRT-PCR of **(C)** miR-128-3p and **(D)** FOXO4 mRNA expression in tumor tissues. **(E)** Western blot and quantification of EMT markers E-cadherin, ZO-1, vimentin, and N-cadherin in tumor tissue. Protein expression was normalized to that of GAPDH. **(F)** Western blot and quantification of TGF-β, SMAD2, and SMAD3 in tumor tissue. Protein expression was normalized to that of GAPDH. **(G)** Western blot and quantification of p-JAK2, JAK2, p-JAK3, JAK3, p-STAT3, and STAT3 in tumor tissue. Phosphorylated protein expression was normalized to that of total proteins. Data are shown as the mean ± SD (*n* = 5); *P < 0.05.

### Exosomal miR-128-3p Expression Was Positively Correlated With Clinical Progression of CRC

From a clinical perspective, we investigated the correlation between exosomal miR-128-3p and the clinicopathological parameters of CRC patients (Table 1). High expression of miR-128-3p was associated with perineural invasion (PNI), lymphovascular invasion (LVI), tumor stage, and CA 19-9 content (*P* < 0.05). Multivariate analysis (Table 2) showed that miR-128-3p expression in CRC patients was associated with tumor stage and PNI levels (*P* < 0.05). These data indicated that the expression of miR-128-3p was higher in patients with later tumor stage (III–IV) and higher PNI level.

**Table 1:** Correlation between exosomal miR-128-3p expression and clinicopathologic parameters of 66 patients with colorectal cancer.

**Parameters**	***n* (%)**	**Exosomal miR-128-3p expression**		
		**Low**	**High**	***P***
Gender				0.641
Male	37 (56.1)	20	17	
Female	29 (43.9)	14	15	
Age, years				0.266
<60	23 (34.8)	14	9	
≥60	43 (65.2)	20	23	
Tumor site				0.143
Colon	31 (47)	13	18	
Rectal	35 (53)	21	14	
Tumor size, cm				0.316
<5	31 (47)	18	13	
≥5	35 (53)	16	19	
Tumor grade				0.397
Poor	8 (12.1)	3	5	
Moderate/Well	58 (87.9)	31	27	
PNI				**<0.001**
Absence	42 (63.6)	29	13	
Presence	24 (36.4)	5	19	
LVI				**<0.001**
Absence	43 (65.2)	29	14	
Presence	23 (34.8)	5	18	
Tumor stage^*^				**<0.001**
I~II	35 (53)	27	8	
III~IV	31 (47)	7	24	
CEA, ng/mL				0.141
<5	43 (65.2)	25	18	
≥5	23 (34.8)	9	14	
CA 19–9, U/mL				**0.002**
<37	18 (27.3)	15	3	
≥37	48 (72.7)	19	29	
Overall	66 (100)	34	32	

* *The 8th edition of the AJCC Cancer Staging Manual; Boldface indicates P < 0.05. PNI, perineural invasion; LVI, lymphovascular invasion; CEA, carcinoembryonic antigen; CA19–9, carbohydrate antigen 19–9*.

**Table 2:** Multivariate analysis of the relationship between exosomal miR-128-3p expression and clinicopathologic parameters.

**Parameters**	**B**	***p***	**OR**	**95% CI**
Presence PNI	2.307	**0.003**	10.044	2.181–46.260
Presence LVI	0.196	0.848	1.217	0.164–9.040
Tumor stage^*^ (III~IV)	2.568	**0.016**	13.041	1.616–105.258
CA 19–9 ≥ 37 (U/mL)	1.780	0.062	5.930	0.912–38.544

* *The 8th edition of the AJCC Cancer Staging Manual; Boldface indicates P < 0.05. PNI, perineural invasion; LVI, lymphovascular invasion; CA19–9, carbohydrate antigen 19-9*.

## Discussion

EMT is an important biological process that plays a critical role in tumor metastasis and is commonly observed in tumor samples from CRC patients (Qi et al., 2014; Guo et al., 2016). However, the precise molecular events that initiate this complex process in CRC are not fully understood. In this study, HCT-116 cells that have undergone EMT secreted exosomes that expressed high levels of miR-128-3p. More importantly, these exosomes enabled the intercellular transfer of pro-EMT characteristics, resulting in the induction of EMT even in normal HCT-116 cells. We propose that this transfer of pro-EMT characteristics between CRC cells was partially mediated by exosomal miR-128-3p, which consequently regulated FOXO4 expression to affect CRC progression.

As important paracrine factors found in many cell types including tumor cells, exosomes have been demonstrated as regulators of cell-to-cell communication and are crucial signaling intermediates for key pathways (Thery, 2015). Exosome biogenesis and endocytosis remain poorly understood, and whether exosomes can specifically recognize their receptor cells requires further exploration (Andaloussi et al., 2013). Pathological microenvironments not only influence the production of exosomes, but also the contents of exosomal cargo including miRNAs (Feng et al., 2014). miRNAs control gene expression patterns by blocking protein translation or inducing mRNA degradation, thereby serving as potential diagnostic markers and therapeutic targets in tumors such as CRC, liver cancer, and ovarian carcinoma (Hur et al., 2013; Vaksman et al., 2014; Qiao et al., 2017). In the current study, subjecting HCT-116 cells to overexpression or silencing of miR-128-3p, a pro-EMT miRNA, yielded corresponding changes in the content of said miRNA in isolated exosomes. The miR-128-3p-overexpressing exosomes were then able to horizontally transfer their cargo to normal HCT-116 cells, inducing EMT via TGF-β/SMAD and JAK/STAT signaling. Consistent with our findings, Cai et al. reported that miR-128-3p was among the most upregulated miRNAs in chemoresistant, metastatic non-small-cell lung cancer cells, and that the effect of miR-128-3p is associated with Wnt/β-catenin and TGF-β activation (Cai et al., 2017). To further confirm the effect of miR-128-3p on EMT in CRC cells, we evaluated the regulatory role of FOXO4, a target of miR-128-3p, on EMT. As anticipated, miR-128-3p-induced EMT was accompanied by the concurrent downregulation of FOXO4, whereas FOXO4 overexpression counteracted the pro-EMT effect of miR-128-3p. These findings are supported by reports in the literature that collectively established the anti-EMT role of FOXO4 in a variety of cancer types, such as gastric cancer (Su et al., 2014) and non-small-cell cancer (Xu et al., 2014; Li et al., 2016).

Inflammatory microenvironments play an important role in cancer progression, and the correlation between inflammation and EMT is a critical factor in understanding tumor metastasis (Suarez-Carmona et al., 2017). We used the inflammatory cytokine IL-6 as a trigger of EMT as it has been demonstrated to promote EMT in a variety of cancer cells (Sullivan et al., 2009; Xiao et al., 2017). Treatment of HCT-116 cells with IL-6 resulted in the activation of TGF-β/SMAD and JAK/STAT3 signaling, which have been implicated in EMT. TGF-β has been reported to regulate the growth, differentiation, and migration of nearly all cell types (Papageorgis, 2015), and multiple factors are associated with TGF-β/SMAD signaling-induced EMT (Jalali et al., 2012; Liu et al., 2016). The activation of TGF-β/SMAD signaling via extracellular vesicles has been demonstrated by Yamada et al., who showed that extracellular vesicles derived from CRC cells were enriched in TGF-β1 and conferred phenotypic alterations in T cells via TGF-β/SMAD activation (Yamada et al., 2016). In addition, inflammation-related autocrine-paracrine events converging in tumor cells typically result in STAT3 activation, which mediates a transcriptional response favoring tumor survival, proliferation, and angiogenesis (Jarnicki et al., 2010). Moreover, abnormalities in the JAK/STAT pathway are involved in CRC oncogenesis, with aberrant and persistent STAT3 activation being a frequent observation in human CRC that is often associated with poor outcome (Spano et al., 2006; Waldner et al., 2012).

We herein showed that exosomal miR-128-3p was horizontally transferred between HCT-116 cells. This delivery successfully caused cellular signaling via downstream responses, including FOXO4 downregulation, enhanced migration and invasion, and TGF-β/SMAD and JAK/STAT3 activation. In other words, the same phenomena caused by overexpression of miR-128-3p in parental cells were apparent in recipient cells, validating the claim that exosomal transfer was an effective route of intercellular communication. It is encouraging that exosomal miR-128-3p-regulated tumor growth and EMT are also validated in xenograft tumor samples.

## Conclusions

Our findings suggested that miR-128-3p is implicated in regulating EMT by directly suppressing its downstream target gene FOXO4 to activate TGF-β/SMAD and JAK/STAT3 signaling. The pro-EMT properties of miR-128-3p could be transferred to neighboring CRC cells via exosomal delivery, further affecting EMT-associated CRC progression. We propose that the effect of the miR-128-3p/FOXO4 cascade on EMT should be highlighted as a potential therapeutic target for combatting CRC.

## Data Availability Statement

The datasets generated for this study are available on request to the corresponding author.

## Ethics Statement

The studies involving human participants were reviewed and approved by internal review and ethics boards of Zhongnan Hospital of Wuhan University. The patients/participants provided their written informed consent to participate in this study. The animal study was reviewed and approved by Model Animal Research Institute at Wuhan Myhalic Biotechnology Co., Ltd.

## Author Contributions

BX conceptualized, designed the study, and critically revised the manuscript. JB, XZ, and DS performed most of the experiments, analyzed the data, and prepared the figures. CY assisted in preparing the figures. QL and SH performed statistical analysis of the data. YF, WZ, and JS collected the clinical data. JB wrote the first draft of the manuscript. XZ, ZX, and SW contributed to the preparation of the manuscript. All authors have read and approved the final version of the mansucript.

## Conflict of Interest

The authors declare that the research was conducted in the absence of any commercial or financial relationships that could be construed as a potential conflict of interest.
